# Construction and Validation of Prediction Model of Severe Abdominal Pain Post-Transarterial Chemoembolization in Patients with HBV-Associated Primary Liver Cancer

**DOI:** 10.1155/2022/5203166

**Published:** 2022-07-30

**Authors:** Yaobo Yang, Sipan Chen, Zhaoyong Yan, Yang Jiao, Xiang Yan, Yulong Li

**Affiliations:** ^1^Department of Interventional Radiology, Shaanxi Provincial People's Hospital, Xi'an, Shaanxi 710068, China; ^2^Department of Hepatobiliary Surgery, Shaanxi Provincial People's Hospital, Xi'an, Shaanxi 710068, China; ^3^Department of Gastroenterology, Shaanxi Provincial People's Hospital, Xi'an, Shaanxi 710068, China

## Abstract

**Objective:**

This study is aimed at constructing and evaluating a prediction model of severe abdominal pain post-transcatheter arterial chemoembolization in patients with HBV-related primary liver cancer.

**Methods:**

Patients with HBV-associated primary liver cancer who received transarterial chemoembolization (TACE) from March 2019 to March 2022 in the Interventional Therapy Department of our hospital were selected as the subjects, and the included 160 patients were randomly divided into modeling group (*n* = 120) and validation group (*n* = 40) in a ratio of 3 : 1. Visual analog scale (VAS) was used to assess pain severity. 120 patients in the modeling group were divided into no/mild abdominal pain group and severe abdominal pain group. The clinical data of the patients, including gender, age, TACE treatment history, vascular invasion, maximum diameter of tumor, infarction degree, preoperative Eastern Oncology Collaboration Group (ECOG) score, and Lipiodol dosage, were analyzed. Receiver operating characteristic (ROC) curve was used to evaluate the predictive value of the prediction model for severe abdominal pain post-TACE.

**Results:**

A total of 116 patients (72.50%) had severe abdominal pain after TACE. Univariate analysis showed that severe abdominal pain after TACE in the modeling group was associated with TACE treatment history, maximum tumor diameter, infarction degree, and preoperative ECOG score (all *P* < 0.05), but not related to gender, age, vascular invasion, and Lipiodol dosage (all *P* > 0.05). Logistic regression analysis showed that TACE treatment history, maximum tumor diameter, infarction degree, and preoperative ECOG score were all independent influencing factors for acute abdominal pain post-TACE in HBV-HCC patients (all *P* < 0.05). The prediction model equation was *Y* = −3.673 + 1.722 × TACE treatment history + 1.175 × tumor maximum diameter + 2.064 × infarction degree + 1.555 × preoperative ECOG score. Goodness-of-fit test results showed no significant difference between the established prediction model and the observed value (*χ*^2^ = 1.645, *P* = 0.560) and *R*^2^ = 0.821, suggesting that the prediction ability of the model was relatively accurate. ROC analysis results showed that the area under the curve (AUC) of severe abdominal pain after TACE was 0.916 (0.862~0.970) and 0.902 (95% CI: 0.841~0.963) in the modeling group and the verification group, respectively.

**Conclusion:**

TACE treatment history, tumor maximum diameter, infarction degree, and preoperative ECOG score are independent influencing factors for severe abdominal pain post-TACE in patients with HBV-HCC, and the prediction model established on this basis has good application value.

## 1. Introduction

Primary liver cancer is one of the most common malignant tumors in China, with 410,000 new cases and 390,000 deaths in 2020, ranking the fourth in the incidence of malignant tumors and adversely affecting the health of Chinese residents, with a 5-year survival rate of only 14.1% [1, 2]. According to pathological characteristics, primary liver cancer can be divided into hepatocellular carcinoma (HCC), intrahepatic cholangiocarcinoma, and mixed HCC-cholangiocarcinoma, among which HCC is the most common, accounting for more than 75% [3]. Among the known causes, chronic hepatitis B, chronic hepatitis C, and nonalcoholic steatohepatitis are the most common causes of primary liver cancer [4, 5]. According to the report, the proportion of liver cancer caused by hepatitis B is as high as 92.05% [6]. With the advancement of surgical treatment, radiotherapy, chemotherapy, immunotherapy, targeted therapy, and liver transplantation, the expected survival and quality of life of HCC patients were significantly improved [7]. However, since most patients with liver cancer have been in the middle-late stage at diagnosis and unable to accept surgery treatment, interventional treatment become one of the main treatment approaches for patients with liver cancer. Interventional therapies include transarterial chemoembolization (TACE) and hepatic arterial infusion chemotherapy (HAIC) [8, 9]. Among them, TACE is widely used. TACE can increase the concentration of chemotherapy drugs exposed to tumors by injecting large doses of chemical drugs locally to the tumor target lesions, promoting tumor embolization infarction or necrosis [10, 11]. Postembolic syndromes, including acute abdominal pain, nausea, and vomiting, are common after TACE, which is an important reason for prolonged hospital stay, decreased treatment effect, and interruption of treatment [12]. At present, clinical studies have reported that the incidence and severity of abdominal pain vary greatly in different cohorts of HCC patients after TACE treatment [13, 14]. This study analyzed the occurrence characteristics of severe abdominal pain in HBV-related primary liver cancer patients in our hospital, explored its influencing factors, and constructed a clinical prediction model, aiming to provide valuable reference for the risk classification of severe abdominal pain in patients, strengthening targeted intervention, and improving pain management.

## 2. Subjects and Methods

### 2.1. Subjects

Patients with HBV-related primary liver cancer who received TACE from March 2019 to March 2022 in the Interventional Therapy Department of our hospital were selected as the study subjects. Inclusion criteria are as follows: (1) primary liver cancer was confirmed by pathology and met the diagnostic criteria [15]; (2) >20 years of age; (3) the tumor was consistent with <70% liver, in line with TACE criteria; (4) no extrahepatic metastasis before surgery, and the estimated survival time > 3 months; (5) HBV-related primary liver cancer; and (6) complete clinical data. Exclusion criteria are as follows: (1) severe abdominal pain before surgery or a history of long-term use of painkillers, (2) complicated with other malignant tumors, (3) non-HBV-related primary liver cancer, (4) abdominal pain caused by complications in addition to TACE, and (5) confused patients such as hepatic encephalopathy. 160 patients meeting the above criteria were randomly divided into the modeling group (*n* = 120) and the validation group (*n* = 40) according to the ratio of 3 : 1. All the subjects in this study signed informed consent for the study, and this study was approved by the medical ethics committee of the hospital.

### 2.2. Pain Assessment

Referring to “Expert Consensus on Pain Management after Adult Surgery” [16], the trained professional physicians of hepatology evaluated the severity of severe abdominal pain at 1 h, 6 h, 12 h, and 24 h after TACE for HBV-HCC patients by using visual analogue scale (VAS) [14]. The assessment tool was a scale without any mark on the patient's surface. The scale of the physician's surface was 1-100 mm, with one end marked with “no pain” and the other marked with “most severe pain.” The corresponding score was obtained according to the pain intensity of the patient. Pain severity assessment is as follows: 0 is no pain; 1 ~ 3 is mild pain, manifested as discomfort, heavy pressure pain, dull pain, etc.; 4 ~ 6 is moderate pain, manifested as jumping pain, burning sensation, spasm, etc.; and 7 ~ 10 is severe pain, which interferes with normal activities. 120 patients in the modeling group were divided into no/mild abdominal pain group and severe abdominal pain group (moderate/severe abdominal pain). During the patient's abdominal pain, an appropriate amount of short-acting analgesics would be used, which were in line with humanistic care and ethics, but the effect of the selected analgesics generally lasted for 4-6 hours, so as not to affect the assessment of abdominal pain at subsequent time points.

### 2.3. Clinical Data Collection

According to the requirement that the variables in the risk factor survey should be 5 ~ 10 times the sample size, this study included 8 variables through previous research reports and clinical practice, including gender, age, TACE treatment history, vascular invasion, tumor maximum diameter, infarction degree, preoperative ECOG score [17], and Lipiodol dosage. All data were obtained through the hospital patient medical record management system. Data entry was performed by two people at the same time to ensure the accuracy of information. Scorings were done by fixed staffs, and the principle of blinding was adopted.

### 2.4. Statistical Analysis

SPSS21.0 was used to analyze the collected experimental data. The measurement data in accordance with the normal distribution were represented by $\overset{¯}{X}\pm S^{\prime }$. The comparison of measurement data between two groups was performed by the group *t-*test. The counting data were represented by the number of cases or rates. The comparison of counting data between two groups was performed by the *χ*^2^ test. The variables with statistical significance in the univariate analysis were assigned and included in the multivariate analysis. Multivariate analysis was conducted by logistic regression model, and ROC curve was used to evaluate the predictive value of the model for predicting severe abdominal pain post-TACE. ROC curve plotting was performed using the GraphPad 6.0 software. The goodness-of-fit test method was used to test the difference between the model established in this study and the actual observation. *P* > 0.05 indicated that the model has good feasibility. *P* < 0.05 was considered statistically significant.

## 3. Results

### 3.1. Features of Severe Abdominal Pain Post-TACE

A total of 116 of 160 patients developed severe abdominal pain after TACE, with an incidence of 72.50%. The duration of pain in patients with severe abdominal pain was 55-220 min, with an average of 125 ± 36 min. The number of patients who scored 4-6 points in VAS at 1 h and 6 h after TACE was relatively high, and the number of patients who scored 1-3 points in VAS at 12 h and 24 h after TACE was relatively high (Table 1).

### 3.2. Comparison of Clinical Data between the Modeling Group and the Validation Group

There were no significant differences between the modeling group and the validation group in gender, age, TACE treatment history, vascular invasion, tumor maximum diameter, infarction degree, preoperative ECOG score, and Lipiodol dosage (all *P* > 0.05, Table 2).

### 3.3. Univariate Analysis of Severe Abdominal Pain Post-TACE in the Modeling Group

Univariate analysis showed that severe abdominal pain post-TACE in the modeling group was associated with TACE treatment history, maximum tumor diameter, infarction degree, and preoperative ECOG score (all *P* < 0.05), but not related to gender, age, vascular invasion, and Lipiodol dosage (all *P* > 0.05, Table 3).

### 3.4. Multivariate Logistic Regression Analysis of the Factors Influencing Severe Abdominal Pain Post-TACE

The significant variables in single-factor analysis, including TACE treatment history, maximum tumor diameter, infarction degree, and preoperative ECOG score, were included in the multivariate regression analysis model. The variables assigning was as follows: TACE treatment history (yes = 1, no = 0), maximum tumor diameter (≥5 cm = 1, <5 cm = 0), infarction degree (complete = 1, incomplete = 0), and preoperative ECOG score (2 = 1, 0- 1 = 0). The final logistic regression analysis results showed that TACE treatment history, maximum tumor diameter, infarction degree, and preoperative ECOG score were all independent factors influencing severe abdominal pain post-TACE in HBV-HCC patients (all *P* < 0.05, Table 4).

### 3.5. Prediction Model Establishment and ROC Evaluation

According to the risk factors in Table 3, the prediction model of severe abdominal pain after TACE was constructed: *P* = 1/(1 + *e*^−*Y*^), where *P* is the probability of severe abdominal pain after TACE, *e* is the natural logarithm, and *Y* = −3.673 + 1.722 × TACE treatment history + 1.175 × maximum tumor diameter + 2.064 × infarction degree + 1.555 × preoperative ECOG score. Goodness-of-fit test results showed that there was no significant difference between the prediction model of severe abdominal pain post-TACE and the observed value (*χ*^2^ = 1.645, *P* = 0.560), and *R*^2^ = 0.821, suggesting that the prediction ability of the model was relatively accurate. ROC analysis results showed that the AUC of severe abdominal pain post-TACE in the modeling group and the verification group was 0.916 (0.862~0.970) and 0.902 (95% CI: 0.841~0.963), respectively (Table 5 and Figure 1).

## 4. Discussion

With the change of living standard and lifestyle, the incidence and mortality of liver cancer are increasing year by year. According to the report of the International Agency for Research on Cancer (IARC), there were 841,000 cases and 781,000 deaths about liver cancer worldwide in 2018 [18, 19]. The incidence and deaths of liver cancer in my country account for more than half of the world, and the proportion of liver cancer in my country caused by hepatitis B is as high as 90% [20]. Currently, for patients with primary liver cancer, TACE is commonly used clinically to block tumor blood supply and deposit chemotherapy drugs around the tumor so as to play a role of local chemotherapy. TACE is carried out 600,000 to 800,000 times per year in China [21]. TACE is helpful to improve the survival benefit of patients with primary liver cancer. However, in clinical practice, severe abdominal pain post-TACE will prolong the hospital stay of patients, affect their postoperative recovery, and even interrupt the treatment in severe cases [22, 23]. In the present study, 116 of 160 patients developed severe abdominal pain after TACE, with an incidence of 72.50%. The duration of pain in patients with severe abdominal pain was 55-220 min, with an average of 125 ± 36 min. The number of patients with 4-6 points in VAS at 1 h and 6 h post-TACE was relatively high, and the number of patients with 1-3 points in VAS at 12 h and 24 h post-TACE was relatively high. These suggested that the incidence of severe abdominal pain was relatively high at the early stage of TACE, and that the number of severe abdominal pain gradually decreased with the increase of time.

Previous studies [24, 25] have found that TACE treatment experience, liver cancer surgery or transplantation history, diabetes, chronic liver disease history, pain history, CRP level, ECOG score, preoperative anxiety, and postoperative TACE are risk factors for severe abdominal pain post-TACE. Severe abdominal pain post-TACE has a high incidence and has many influencing factors, so it is particularly important to actively prevent abdominal pain. Multivariate logistic regression analysis of this study showed that TACE treatment history, maximum tumor diameter, infarction degree, and preoperative ECOG score were independent risk factors for the occurrence of severe abdominal pain post-TACE. Specifically, the larger the tumor diameter is, the more embolization agents such as Lipiodol are used in TACE, and the greater the tumor embolization degree is, the more severe the abdominal pain reaction caused by ischemic necrosis in a short period of time [26]. However, patients with a history of TACE are relatively less sensitive to repeated same irritant pain. Research [27, 28] shows that patients with a history of TACE are 7.931 times more sensitive to abdominal pain than those without TACE, which is similar to the results of the present study. The higher the ECOG score, the more advanced or larger the liver cancer of the patient is, and the more embolic agents such as Lipiodol used in TACE are correspondingly larger, resulting in more severe abdominal pain.

In this study, prediction model was established. The AUC of severe abdominal pain after TACE in the modeling group and the validation group was 0.916 (0.862~0.970) and 0.902 (95% CI: 0.841~0.963), respectively, indicating that the prediction model established in this study had a high predictive value for severe abdominal pain post-TACE. At present, severe abdominal pain post-TACE has a high incidence and has certain subjectivity with the existence of misdiagnosis and missed diagnosis. The present model can directly predict the risk factors of severe abdominal pain post-TACE without the influence of blood environment and exogenous factors. The application of this model combined with clinical indicators can improve the sensitivity of diagnosis and help patients to detect severe abdominal pain post-TACE at an early stage, so that treatment and control measures can be adopted as soon as possible to avoid further development and aggravation of the disease.

In conclusion, severe abdominal pain post-TACE is associated with multiple factors including TACE treatment history, maximum tumor diameter, infarction degree, and preoperative ECOG score. In this study, the logistic regression risk prediction model of postoperative severe abdominal pain post-TACE established based on the above factors has a good prediction effect, and clinical intervention can be carried out according to the above risk factors to reduce the incidence of postoperative severe abdominal pain. However, this study also has shortcomings such as small sample size and only the visual analog scale (VAS) used to assess the severity of pain. In the future, the research sample can be further expanded, and multiple means of assessing pain severity can improve the reliability of the study to provide more support for clinical application.

## Figures and Tables

**Figure 1:** ROC analysis of the model's predictive value in predicting severe abdominal pain in the modeling group and validation group.

**Table 1:** Features of severe abdominal pain post-TACE (VAS, points (%)).

Timing	0 points	1 ~ 3 points	4 ~ 6 points	7 ~ 9 points	10 points
1 h	3 (1.88)	21 (13.13)	100 (62.50)	26 (16.25)	10 (6.25)
6 h	7 (4.38)	43 (26.88)	83 (51.88)	27 (16.88)	6 (3.75)
12 h	13 (8.13)	66 (41.25)	62 (38.75)	19 (11.88)	0 (0.00)
24 h	19 (11.88)	82 (51.25)	53 (33.13)	6 (3.75)	0 (0.00)

**Table 2:** Comparison of clinical data between the modeling group and the validation group.

Factor	Classification	Modeling group (*n* = 120)	Validation group (*n* = 40)	*χ* ^2^ value	*P* value
Gender	Male	65	25	0.847	0.358
	Female	55	15		

Age (years)	≥60	43	18	1.069	0.301
	<60	77	22		

TACE treatment history	Yes	46	17	0.218	0.640
	No	74	23		

Vascular invasion	Yes	62	23	0.410	0.522
	No	58	17		

Maximum diameter of tumor (cm)	<5	75	27	0.325	0.569
	≥5	45	13		

Infarction degree	Incomplete	103	33	0.261	0.609
	Complete	17	7		

Preoperative ECOG score (points)	0 ~ 1	99	30	1.080	0.299
	2	21	10		

Lipiodol dosage (mL)	<10	86	28	0.041	0.840
	≥10	34	12		

**Table 3:** Univariate analysis of severe abdominal pain post-TACE in the modeling group.

Factor	Classification	No/mild abdominal pain group (*n* = 35)	Severe abdominal pain group (*n* = 85)	*χ* ^2^ value	*P* value
Gender	Male	20	45	0.176	0.675
	Female	15	40		

Age (years)	≥60	13	30	0.037	0.848
	<60	22	55		

TACE treatment history	Yes	5	41	12.091	<0.001
	No	30	44		

Vascular invasion	Yes	22	40	2.478	0.116
	No	13	45		

Maximum diameter of tumor (cm)	<5	7	38	6.456	0.011
	≥5	28	47		

Infarction degree	Incomplete	1	16	5.198	0.023
	Complete	34	69		

Preoperative ECOG score (points)	0 ~ 1	33	66	4.754	0.029
	2	2	19		

Lipiodol dosage (mL)	<10	10	24	0.001	0.970
	≥10	25	61		

**Table 4:** Multivariate logistic regression analysis of the factors influencing severe abdominal pain post-TACE.

Risk factor	*Β* value	SE value	Ward value	OR value	95% CI	*P* value
TACE treatment history	1.722	0.631	7.443	5.593	1.624~ 19.265	0.016
Maximum tumor diameter	1.175	0.583	4.055	3.235	1.032~ 1.142	0.035
Infarction degree	2.064	0.672	9.437	7.880	2.111~ 29.413	<0.001
Preoperative ECOG score	1.555	0.615	6.391	4.734	1.418~ 15.803	0.023

**Table 5:** Prediction model establishment and ROC evaluation.

Index	AUC	Sensitivity (%)	Specificity (%)	95% CI	Standard error	*P* value
Modeling group	0.916	90.10	87.16	0.862~0.970	0.028	<0.001
Validation group	0.902	89.67	86.55	0.841~0.963	0.031	<0.001

## Data Availability

The labeled datasets used to support the findings of this study are available from the corresponding author upon request.
